The article "Blueberry juice protects osteocytes and bone precursor cells against oxidative stress partly through SIRT1" was published in 2019. Journal: FEBS Open Bio.

# Blueberry juice protects osteocytes and bone precursor cells against oxidative stress partly through SIRT1

**DOI:** 10.1002/2211-5463.12634

**Published:** 2019-04-20

**Authors:** Vladana Domazetovic, Gemma Marcucci, Federica Pierucci, Gennaro Bruno, Lorenzo Di Cesare Mannelli, Carla Ghelardini, Maria Luisa Brandi, Teresa Iantomasi, Elisabetta Meacci, Maria Teresa Vincenzini

**Affiliations:** ^1^ Department of Biomedical Experimental and Clinical Sciences ‘Mario Serio’ University of Florence Italy; ^2^ Department of Health Sciences University of Florence Italy; ^3^ Department of Neuroscience, Psychology, Drug Research and Child Health (NEUROFARBA) Pharmacology and Toxicology Section University of Florence Italy

**Keywords:** antiosteoclastogenic factors, antioxidant activity, apoptosis, blueberry, osteocyte, SIRT1

## Abstract

Oxidative stress and abnormal osteocyte apoptosis are often related to dysregulation of bone turnover and chronic bone loss, and so fruit and vegetables with high antioxidant potential may play an important role in the prevention and/or management of osteoporosis. Osteocytes are the main regulators of bone remodelling. For the first time, we demonstrate here that blueberry juice (BJ), obtained from *Vaccinium myrtillus*, rich in polyphenols, shows antioxidant and antiosteoclastogenic properties in MLO‐Y4 osteocytes. We report that BJ prevents oxidative stress‐induced apoptosis and reverses the increase in receptor activator of nuclear factor κB ligand and sclerostin expression, crucial factors for osteoclast activation and bone resorption. BJ is also able to prevent oxidative stress‐induced cell cytotoxicity in bone marrow mesenchymal stromal cells (MSCs), which are considered to be an important tool for cell therapy in bone disorders. No significant difference in preventing these events was observed between BJ and blueberry dry extract containing equal amounts of total soluble polyphenols. We have also shown that blueberry acts as both an antioxidant and an activator of sirtuin type 1, a class III histone deacetylase involved in cell death regulation and considered a molecular target for blocking bone resorption without affecting osteoclast survival. Overall, these novel data obtained in osteocytes and MSCs may help us clarify the mechanisms by which blueberry counteracts oxidative stress‐induced damage in bone remodelling and osteogenesis at the cellular and molecular level. Our findings are consistent with the reported beneficial effects of blueberry on bone tissue reported in animal studies, which suggest that blueberry may be a useful supplement for the prevention and/or management of osteoporosis and osteogenic process.

The article "Blueberry juice protects osteocytes and bone precursor cells against oxidative stress partly through SIRT1" was published in 2019. Journal: FEBS Open Bio.

**Abbreviations**
Ac‐p53: acetylated‐p53
BB: blueberry
BE: blueberry dry extract
BJ: blueberry juice
ERK1/2: extracellular signal‐regulated kinase 1/2
FBS: fetal bovine serum
H_2_DCFDA: 2′,7′‐dichlorodihydrofluorescein diacetate
JNK: c‐Jun N‐terminal kinase
MSC: marrow mesenchymal stromal cell
MTT: 3‐(4,5‐dimethylthiazol‐2‐yl)‐2,5‐diphenyl‐tetrazolium bromide
NBT: Nitroblue tetrazolium
PARP‐1: poly‐(ADP‐ribose) polymerase 1
RANKL: receptor activator of nuclear factor κB ligand
ROS: reactive oxygen species
SIRT1: sirtuin type 1
TSP: total soluble polyphenols

Fruits and vegetables rich in phytochemicals, such as phenolic acids, are essential for bone formation and health 1, 2, 3, and their daily consumption may be important in increasing the bone mass peak 4, 5. These antioxidant compounds scavenge reactive oxygen species (ROS) and reduce oxidative stress in many diseases 3, 5, 6 including bone diseases and, in particular, osteoporosis 7, 8, 9. This latter disease is mainly due to abnormal activation of osteoclasts, inhibition of osteoblast activity and an increase of osteocyte apoptosis due to oxidative stress, which may be the result of oestrogen deficiency and/or other bone diseases 10, 11, 12. Indeed, redox balance regulation in bone cells affects bone turnover and remodelling 13, 14, 15, and microdamage, oxidative stress, and abnormal osteocyte apoptosis are related to an imbalance of the remodelling process with the consequent altered bone formation and a decrease in mineral density 16, 17, 18. The osteocytes are in close contact with the blood flow and contribute to the transfer of endogenous and exogenous compounds to osteoblasts and osteoclasts, regulating their formation and activity 16, 19. Moreover, increased production of ROS damages stem cell self‐renewal and differentiation toward tissue‐specific lineages including bone tissue 20, 21, 22, 23. Given their antioxidant activity, natural polyphenols act as powerful modulators of mesenchymal stromal stem cells, which are considered a useful tool for studying bone regeneration processes and bone tissue engineering treatments 20, 21, 24. Effectively, nutritional approaches to antioxidant strategies can be useful for the treatment and the prevention of bone loss 1, 2, 3, 4, considering the possible adverse side effects associated with anti‐resorptive drugs, such as bisphosphonate or oestrogen therapy. In fact, these therapies reduce significantly bone loss and the osteoclastogenesis but do not restore a normal bone remodelling process 14, 25. In view of this, there is a rising demand for use of natural products as adjuvant therapy or supplementation in combination with medical therapy to promote the restoration of normal bone metabolism. However, there are few data that correlate the antioxidant properties of plants containing bioactive phytochemicals to molecular mechanisms of biological processes involved in the modulation and regulation of bone formation and regeneration in the condition of oxidative stress. In particular, no data are reported on the protective effects of blueberry (BB) phytochemicals against oxidative stress‐induced damage on osteocyte activity and on bone precursor cell viability. Indeed, we previously demonstrated in a murine osteocyte‐like cell line, MLO‐Y4, with similar phenotype and many characteristics of mature osteocytes 26, 27, that thiol antioxidants such as glutathione, *N*‐acetylcysteine and lipoic acid prevent and down‐regulate both apoptosis and osteoclastogenic factors induced by intracellular oxidative stress 18. BBs and, in particular, *Vaccinium mirtillus*, contain high concentrations of well‐characterized anthocyanins, phenolic acids, coumarins, flavonols, flavanols, and phenolic compounds with antioxidant activity 28, 29. Recently, a role for the bioactive compounds contained in *Vaccinium mirtillus* as ‘functional food' for dietary supplementation has been suggested 28, 29. Studies on animal and cell models reveal a positive association of high intake of BB polyphenols with antioxidant properties and high bone mass 30. Indeed, diet‐derived phenolic acids promote bone growth and regulate osteoblast and adipocyte lineage commitment and differentiation in young mice 2, 23, and diets containing BBs prevent osteoporosis in ovariectomized rats 31, 32. However, the molecular mechanisms through which these act are still little known.

The article "Blueberry juice protects osteocytes and bone precursor cells against oxidative stress partly through SIRT1" was published in 2019. Journal: FEBS Open Bio.

The aim of this study was to evaluate the ability of natural compounds contained in BB juice (BJ) and BB dry extract (BE) to preserve osteocyte activity and bone precursor cell regeneration in the presence of oxidative stress, and to identify possible biological mechanisms and targets on which BB phytochemicals can act to stimulate bone formation and to maintain normal bone remodelling in bone diseases related to oxidative stress. For this study, MLO‐Y4 osteocyte‐like cells and bone mesenchymal stromal stem cells (MSCs) were used. MLO‐Y4 constitutes a model to study *in vitro* osteocyte viability and apoptosis in response to microdamage and bone diseases 26, 27, 33, whereas MSCs are considered an important tool for cell therapy in bone disorders due to their ability to differentiate into various tissues including bone tissue 20, 21.

The results demonstrate both in osteocytes and in MSCs, cultured in serum deprivation, that BJ and BE are able to reduce ROS levels and to prevent apoptosis and cytotoxicity due to oxidative stress. Moreover, in starved osteocytes they prevent the up‐regulation of receptor activator of nuclear factor κB ligand (RANKL) and sclerostin, osteoclastogenic factors related to apoptosis and bone resorption. The effects of BJ and BE are in part mediated by activity of SIRT1, which has been proposed as a potential target to restore a normal bone remodelling process and for anabolic therapies against excessive bone resorption in osteoporosis.

The article "Blueberry juice protects osteocytes and bone precursor cells against oxidative stress partly through SIRT1" was published in 2019. Journal: FEBS Open Bio.

## Results

### Effect of BJ and BE on ROS production in starved MLO‐Y4 cells and in cell‐free model

In MLO‐Y4 cells, oxidative stress was induced by serum deprivation (starved cells), and two different BB preparations, BJ and BE, were used given that BBs are commercialised in different ways, mainly as fresh or frozen products but also as juice or dry extract. Previously, we demonstrated a remarkable increase of ROS after 4 and 24 h in starved MLO‐Y4 cells 18, as reported in the present study in Fig. 1A. In these experimental conditions, the antioxidant effect of BJ containing various concentrations (from 7.5 to 60 μg·mL^−1^) of total soluble polyphenols (TSP) was measured. Figure 1A shows that the lowest concentrations (7.5–15 μg·mL^−1^) reduced significantly ROS levels after 4 h by about 25% and the highest concentrations (30–60 μg·mL^−1^) by about 50%, as compared to starved cells. ROS reduction elicited by BJ treatments after 24 h significantly and gradually increased from 25% to 50%, reaching the maximum effect at 30 μg·mL^−1^ TSP (Fig. 1A). Next, we compared the BJ antioxidant effect to that of BE at this concentration of TSP. As shown in Fig. 1B, no difference was observed between BJ and BE after both 4 and 24 h of treatment. Effectively, BJ and BE also showed a similar antioxidant capacity when superoxide anion radical scavenging activity was measured in a cell‐free model using the same concentration of TSP (30 μg·mL^−1^) (Fig. 1C).

**Figure 1:** Antioxidant effect of BJ and BE on intracellular ROS in MLO‐Y4 cells and in a cell‐free model. (A,B) Intracellular ROS, detected by measuring the fluorescence intensity of the probe 2′,7′‐dichlorodihydrofluorescein diacetate (H_2_ DCFDA), were measured in MLO‐4Y cells cultured for 4 and 24 h in complete medium (C, control) or in serum‐free medium (S, starved cells). Starved cells were treated or not with BJ at various concentrations (μg·mL^−1^) of total soluble polyphenols (TSP) (A), or with 30 μg·mL^−1^ TSP of BJ or BE (B), as reported in Materials and methods. (C) The xanthine/xanthine oxidase system was used for $O_{2}^{-\cdot }$ production and nitroblue tetrazolium (NBT) was used as target for the detection of scavenging activity of $O_{2}^{-\cdot }$ by BJ and BE in a cell‐free model, as reported in Materials and methods. In (A,B), ROS data, normalized on total protein content, are expressed as fold‐increase over the respective control values and are the mean ± SEM of four experiments performed in duplicate. In (C), $O_{2}^{-\cdot }$ scavenging activity is expressed as absorbance arbitrary units (A.U.) and the data are the mean ± SEM of three experiments performed in duplicate. Data were evaluated by using one‐way ANOVA followed by Bonferroni's *post hoc* test. ^□^ *P* ≤ 0.001 compared to 4 h untreated starved cells; *P ≤ 0.05; **P ≤ 0.001 compared to the respective untreated starved cells; ^○^ *P* ≤ 0.05 compared to 30 and 60 μg·mL^−1^ TSP treated cells; ^∆^ *P* ≤ 0.05 compared to 24 h 7.5 μg·mL^−1^ TSP treated cells; ^●^ *P* ≤ 0.01 compared to control cells.

The article "Blueberry juice protects osteocytes and bone precursor cells against oxidative stress partly through SIRT1" was published in 2019. Journal: FEBS Open Bio.

### Effect of BJ and BE on oxidative stress‐induced RANKL and sclerostin expression and apoptosis in starved MLO‐Y4 cells

The effect of BJ and BE on oxidative stress‐induced overexpression of osteoclastogenic factors, such as RANKL and sclerostin, was investigated. Figure 2A shows that RANKL and sclerostin up‐regulation due to oxidative stress in starved MLO‐Y4 cells 18 was prevented by the treatment with 30 μg·mL^−1^ TSP of BJ or BE, the concentration at which the maximum antioxidant effect was obtained. Since RANKL and sclerostin overexpression have been correlated to c‐Jun N‐terminal kinases (JNK) and extracellular signal‐regulated kinases 1/2 (ERK1/2) activation 18, we evaluated the effect of BJ and BE on the oxidative stress‐induced activation of these kinases. Phosphorylation of both JNK and ERK1/2 was significantly reduced confirming the ability of BJ and BE to counteract these effects (Fig. 2B). Cell apoptosis, induced by oxidative stress after 24 h of starvation as previously reported 18, was assayed by detecting oligonucleosomes and phosphatidylserine on the external surface of the plasma membrane. Both methods of analysis showed that the treatment with 30 μg·mL^−1^ TSP of BJ or BE significantly prevented apoptosis, which decreased by about 70–80% as compared to starved cells (Fig. 3A,B). The protective effect was confirmed by the decrease of 17 kDa caspase‐3 active form that derives from proteolytic cleavage of inactive 32 kDa procaspase‐3 induced by oxidative stress (Fig. 4A). Similarly, the levels of cleaved poly‐(ADP‐ribose) polymerase 1 (PARP‐1), a natural substrate of caspase‐3, decreased in cells treated with BJ or BE (Fig. 4B). Altogether, these results show that BB treatments are effectively able to prevent osteocyte apoptosis.

**Figure 2:** Effect of BJ and BE on RANKL and sclerostin expression, and JNK and ERK phosphorylation in MLO‐Y4 cells. RANKL and sclerostin expression, and ERK and JNK phosphorylation were measured in MLO‐Y4 cells cultured for 24 h in complete medium (C, control) or in serum‐free medium (S, starved cells). Starved cells were treated or not with 30 μg·mL^−1^ of total soluble polyphenols (TSP) of BJ and BE, as reported in Materials and methods. RANKL and sclerostin (A), p‐ERK and p‐JNK (B) were measured by western blot analysis and values are normalized with β‐actin, ERK and JNK bands obtained by densitometric analysis, respectively. Blots are representative of four experiments and data, expressed as fold‐increase over the respective control, are reported as mean ± SEM at the bottom. Data were evaluated by using one‐way ANOVA followed by Bonferroni's *post hoc* test. *P ≤ 0.01; **P ≤ 0.001 compared to the respective control, BJ‐ and BE‐treated cells.

The article "Blueberry juice protects osteocytes and bone precursor cells against oxidative stress partly through SIRT1" was published in 2019. Journal: FEBS Open Bio.

**Figure 3:** Effect of BJ and BE on apoptosis in MLO‐Y4 cells. Apoptosis was measured in MLO‐4Y cells cultured for 24 h in complete medium (C, control) or in serum‐free medium (S, starved cells). Starved cells were treated or not with 30 μg·mL ^−1^ of total soluble polyphenols (TSP) of BJ and BE, as reported in Materials and methods. Apoptosis data, relative to mono‐ and oligonucleosomes released into the cytoplasmic fraction from 10^4^ cells (A), or relative to phosphatidylserine on the external plasma membrane (B), are expressed as fold‐increase over control values and are the mean ± SEM of four experiments performed in duplicate. Data were evaluated by using one‐way ANOVA followed by Bonferroni's *post hoc* test. *P ≤ 0.05 compared to the respective control cells; **P ≤ 0.001 compared to the respective control, BJ‐ and BE‐treated cells.

**Figure 4:** Effect of BJ and BE on active 17 kDa caspase‐3 and PARP‐1 cleavage in MLO‐Y4 cells. Active 17 kDa caspase‐3 and PARP‐1 cleavage were measured in MLO‐4Y cells cultured for 24 h in complete medium (C, control) or in serum‐free medium (S, starved cells) by western blot analysis. Starved cells were treated or not with 30 μg·mL ^−1^ of total soluble polyphenols (TSP) of BJ and BE, as reported in Materials and methods. Densitometric analysis of active 17 kDa caspase‐3 (A) and cleaved PARP‐1 (B) values were normalized with β‐actin bands. Blots are representative of three experiments and data, expressed as fold‐increase over control, are reported as mean ± SEM at the bottom. Data were evaluated by using one‐way ANOVA followed by Bonferroni's *post hoc* test. *P ≤ 0.001; **P ≤ 0.05 compared to the respective control, BJ‐ and BE‐treated cells.

### Involvement of SIRT1 in antiosteoclastogenic and antiapoptotic effect of BJ and BE in starved MLO‐Y4 cells

This study investigated also the role of sirtuin type 1 (SIRT1), a class III histone deacetylase involved in the regulation of apoptosis 34 and activated in mammals by dietary blueberry 35, 36. Figure 5A shows that in our experimental conditions the starvation did not affect SIRT1 expression, which, on the contrary, was remarkably increased by BJ or BE treatment as compared to control and starved cells. Subsequently, SIRT1 activity was investigated by measuring levels of acetylated‐p53 (Ac‐p53), a substrate of SIRT1 also involved in the apoptotic event 34. As reported in Fig. 5B, BJ or BE was able to decrease Ac‐p53 levels as compared to starved cells. This effect was removed completely by EX527, a specific inhibitor of SIRT1, at the concentration able to inhibit SIRT1 activity 37. The involvement of SIRT1 in an antiosteoclastogenic and antiapoptotic effect elicited by BJ and BE was determined in MLO‐Y4 cells transfected with specific SIRT1 siRNA or in the presence of EX527. Figure 5C shows SIRT1 decrease in control cells after 24 h of transfection. SIRT1 down‐regulation induced a significant increase in RANKL, sclerostin and apoptosis levels in 24‐h‐starved cells treated with BJ or BE (Fig. 5D,E). Similarly, SIRT1 inhibition due to EX527 increased apoptosis in starved MLO‐Y4 cells (Fig. 5E).

The article "Blueberry juice protects osteocytes and bone precursor cells against oxidative stress partly through SIRT1" was published in 2019. Journal: FEBS Open Bio.

**Figure 5:** Effect of SIRT1 on RANKL and sclerostin expression and apoptosis in MLO‐Y4 cells treated with BJ and BE. SIRT1 expression (A,C) and Ac‐p53 levels (B) were determined in MLO‐4Y cells in the absence or in the presence of 10 μm EX527. RANKL and sclerostin expression and apoptosis were measured in cells transfected with SIRT1 siRNA or Scr siRNA (D,E) or in the presence of 10 μm EX527 (E). Cells were cultured for 24 h in complete medium (C, control) or in serum‐free medium (S, starved cells). Starved cells were treated or not with 30 μg·mL ^−1^ of total soluble polyphenols (TSP) of BJ and BE, as reported in Materials and methods. Ac‐p53, RANKL and sclerostin levels were measured by western blot analysis and values are normalized with β‐actin bands obtained by densitometric analysis, and blots are representative of three experiments. Apoptosis data were relative to mono‐ and oligonucleosomes released into the cytoplasmic fraction from 10^4^ cells. The data are expressed as fold‐increase over control or starved cell values and are the mean ± SEM of three experiments performed in duplicate. Data were evaluated by using one‐way ANOVA followed by Bonferroni's *post hoc* test. *P ≤ 0.001 compared to BJ‐ and BE‐treated cells without EX527 or with Scr siRNA; ^○^ *P* ≤ 0.01 compared to the respective untreated starved cells with EX527 or with SIRT1 siRNA; ^∆^ *P* ≤ 0.001 compared to untreated starved cells.

The article "Blueberry juice protects osteocytes and bone precursor cells against oxidative stress partly through SIRT1" was published in 2019. Journal: FEBS Open Bio.

### Effect of BJ on ROS production and viability in serum‐deprived MSCs

Since bone formation requires the recruitment, proliferation and osteogenic differentiation of mesenchymal progenitors, we extended our investigation to MSCs. In particular, we investigated the antioxidant ability of BJ and its protective effect against oxidative stress‐reduced viability of MSCs. The antioxidant effect of BJ, containing various concentrations of TSP (7.5–30 μg·mL^−1^), was tested in MSCs cultured for 24 h in the presence of reduced concentrations of serum (0.1%, 0.5%) in order to promote oxidative stress. Indeed, as reported in Fig. 6, serum deprivation determined an increase of ROS production as compared to cells incubated in medium with 10% fetal bovine serum (FBS). A significant ROS increase was also observed in cells cultured with 0.1% FBS as compared to values from cells cultured in 0.5% FBS (Fig. 6A). In the presence of 0.5% FBS, BJ treatment (7.5–30 μg·mL^−1^ TSP) reduced significantly ROS levels at all concentrations used, and 30 μg·mL^−1^ TSP reduced ROS levels to about 70% as compared to untreated cells (Fig. 5A). A similar effect was also obtained in cells cultured in 0.1% FBS (Fig. 6A). The decrease of serum content also induced changes in cell morphology and density (Fig. 6B), and the decrease of cell viability was significantly related to serum deprivation (Fig. 6C).

**Figure 6:** Effect of serum deprivation and BJ on intracellular ROS production, morphology and cell viability in MSCs. MSCs were cultured for 24 h in growth medium with 10%, 0.5%, 0.1% or no FBS, and treated or not with various concentrations of total soluble polyphenols (TSP) of BJ, as reported in Materials and methods. (A) Intracellular ROS production was detected as described in Figure 1 and the data are expressed as fold‐increase over values obtained in cells cultured in 10% FBS. (B) Morphological images of MSCs representative of at least three independent experiments; scale bar: 25 μm. (C) Cell viability was detected by 3‐(4,5‐dimethylthiazol‐2‐yl)‐2,5‐diphenyl‐tetrazolium bromide (MTT) and the absorbance values are reported as arbitrary units (A.U.) from 10^4^ cells. The data are the mean ± SEM of three experiments performed in triplicate. Data were evaluated by using one‐way ANOVA followed by Bonferroni's *post hoc* test. *P ≤ 0.05 compared to cells grown in 10% FBS; ^○^ *P* ≤ 0.05 compared to cells grown in 0.5% or 0.1% FBS without BJ TSP.

Since the incubation of MSCs in a medium containing 0.1% FBS promoted an extensive cell death, leading to a 4‐fold increase of the sub‐G_0_/G_1_ fraction as compared to cells with 10% FBS (4.5 ± 0.1% versus 1.02 ± 0.08%, *n* = 4, *P* < 0.05), the ability of BJ to counteract cell damage was determined in MSCs cultured in 0.5% FBS in which the reduction of the sub‐G_0_/G_1_ fraction was only 2‐fold (2.5 ± 0.2% versus 1.02 ± 0.08%, *n* = 4, *P* < 0.05). As shown in Fig. 6C, BJ (15–30 μg·mL^−1^ TSP) was able to preserve cell viability by approximately 75% as compared with untreated cells, whereas surprisingly, a higher concentration of TSP (60 μg·mL^−1^) did not have a similar protective effect.

The article "Blueberry juice protects osteocytes and bone precursor cells against oxidative stress partly through SIRT1" was published in 2019. Journal: FEBS Open Bio.

### Effect of BJ on cytotoxicity and involvement of SIRT1 in serum‐deprived MSCs

Next, we evaluated the role of SIRT1 in BJ's ability to prevent MSC cytotoxicity. MSCs were incubated with 30 μg·mL^−1^ TSP of BJ and in serum‐deprived medium (0.5% FBS) in the absence or in the presence of EX527 for 24 h. As shown in Fig. 7A, a significant reduction of cytotoxicity (of about 40%) was observed in the presence of BJ TSP compared to untreated cells. Notably, similarly to what observed in osteocytes, the pharmacological inhibition of SIRT1 prevented the protective effect elicited by BJ (Fig. 7A), suggesting the involvement of this deacetylase activity also in these progenitor cells. On the other hand, while the expression of SIRT1 was induced by BJ in MLO‐Y4 cells (Fig. 5A), the protein expression was not changed by BBs in these cells (Fig. 7B).

**Figure 7:** Effect of SIRT1 on toxicity in MSCs treated with BJ. (A) Cell cytotoxicity was determined in MSCs cultured for 24 h in 0.5% FBS in the absence or in the presence of 30 μg·mL ^−1^ of total soluble polyphenols (TSP) of BJ and with or without 10 μm EX527, as reported in Materials and methods. The absorbance values are expressed as arbitrary units (A.U.) from 10^4^ cells and are the mean ± SEM of four experiments performed in quadruplicate. (B) SIRT1 expression was determined by western blot analysis and values are normalized with β‐actin bands obtained by densitometric analysis. Blots are representative of three experiments. Data were evaluated by using one‐way ANOVA followed by Bonferroni's *post hoc* test. *P ≤ 0.05 compared to cells grown in 0.5% FBS; ^°^ *P* ≤ 0.05 compared to cells grown in 0.5% FBS with TSP and without EX527.

## Discussion

The consumption of BBs is considered an important contribution to the diet; this is due to the abundance of various classes of polyphenolic compounds that make this fruit rich in anti‐inflammatory, anti‐hypertensive, antimicrobial, and anticancer properties 29. Studies on bioavailability of BB polyphenols show that some of these are absorbed and present in human plasma for a variable period after intake. In fact, plasma concentrations of many of these compounds increase significantly following the administration of diets containing blueberries, although many of the phytochemicals are modified after absorption 38, 39, 40. Plasma kinetic profiles of BB polyphenols for 2 h after a BJ or BB smoothie intake have been reported 41. Some orally administrated polyphenols, such as anthocyanins or cyanidins, can be absorbed as glycosides and/or aglycones in intact form and as such they are found in the blood 42, 43, 44. Nevertheless, many studies evidence that intake amount, chemical structure, enterohepatic circulation and other individual factors, such as age, gender, gut microbiota, and genetic polymorphisms, play a role in BB polyphenol bioavailability evidencing a complex metabolic fate of these compounds not necessary involving the loss of their function 45, 46.

The article "Blueberry juice protects osteocytes and bone precursor cells against oxidative stress partly through SIRT1" was published in 2019. Journal: FEBS Open Bio.

Among the bioactive substances present in BBs, flavonoids, specifically anthocyanins, have been proven to have a strong antioxidant capacity 28, 29, 30, 40. In this study, the effect of BBs was evaluated in starved MLO‐Y4 cells, a condition that mimics *in vitro* a metabolic situation of oxidative stress that may be similar to what occurs *in vivo* in the bone environment after microdamage and oestrogen deficiency 12, 14, 18, 26, 47. Previously, it has been demonstrated that oxidative stress‐induced apoptosis by starvation in MLO‐Y4 cells is involved in the up‐regulation of osteoclastogenic factors 18. In fact, thiol antioxidants inhibit ROS production due to starvation and prevent both apoptosis and the increase of osteoclastogenic factors. A relationship among these events has been found 18. The present study demonstrates for the first time in MLO‐Y4 cells the antioxidant, antiapoptotic and anti‐osteoclastogenic properties of both BJ and BE containing equal amounts of TSP. In particular, BJ promotes a concentration‐dependent antioxidant effect after 24 h of starvation. Moreover, a similar antioxidant effect between BJ and BE is found in both a cellular and a cell‐free model. This indicates that BB effects are independent of the type of preparation (juice or extract) containing the same TSP amount. Like in starved MLO‐4Y cells, BJ shows the same antioxidant activity also in MSCs cultured at low serum concentrations, a condition that induces intracellular oxidative stress in these cells.

We speculate that the beneficial antioxidant effect of BBs is mainly due to the polyphenolic fraction; in fact, dietary antioxidant polyphenols activate osteoblast function promoting bone growth and inhibiting osteoclast differentiation 1, 2, 3, 4, 5, 31, 32. Literature data show that ROS might be involved in the pathogenesis of bone loss and that nutritional approaches to antioxidant strategies may prevent this 2, 6, 12, 14. Indeed, dietary BBs protect against ovariectomized‐induced osteoblast death 31 and regulate osteoblast differentiation 2. This agrees with the preventive effect of BJ and BE on oxidative stress‐induced up‐regulation of RANKL and sclerostin and osteocyte apoptosis, and this preventive effect occurs by reducing significantly ROS‐induced JNK and ERK1/2 activation present in starved MLO‐4Y cells, as previously reported 18, 41. It has been reported that the up‐regulation of RANKL and sclerostin occurs in osteocytes under various conditions, including bone pathological alterations 12, 16, 19. In fact, RANKL increases osteoclast differentiation and bone resorption, whereas sclerostin, specifically produced in mature osteocytes, is a negative regulator of Wnt/β‐catenin signalling that inhibits osteoblast activity and osteogenesis 16, 48. Our data regarding the down‐regulation of RANKL expression by BJ and BE agree with the inhibitory effect of polyphenol extracts on increased RANKL expression in response to tumour necrosis factor‐α‐induced oxidative stress 4. However, no data are reported on the regulation of sclerostin expression in osteocytes by polyphenols or plant extracts. It is interesting that the effects observed on the osteoclastogenic factors in osteocytes are obtained using concentrations of TSP similar to the polyphenol concentrations of dried plums, which suppress RANKL expression and enhance osteoblast activity 49. The ability of BJ and BE to protect osteocytes from apoptosis is very important considering that abnormal osteocyte apoptosis is closely related to the expression of osteoclastogenic factors and high bone turnover, both events involved in bone loss and osteoporosis 14, 16, 17. Indeed, in young rats fed a diet containing different amounts of BB (from 1% to 10%) there is a significant increase in bone mass and inhibition of osteoclast differentiation associated to RANKL and related to amounts of administered BBs 50. Moreover, polyphenol‐derived phenolic acid present in serum from BB diet‐fed rats is bioactive, stimulating osteoblast differentiation and bone mineralization through Wnt signalling 2, 23. Previous data demonstrated that in MLO‐Y4 cells, starvation‐induced apoptosis is closely related to increased mitochondrial ROS production, which, through JNK activity, induces caspase‐3 activation 18, 47. Furthermore, this study demonstrates that the antiapoptotic ability (apoptosis reduction of about 70–80%) of BJ and BE is higher than their antioxidant capacity (ROS reduction of about 50%). This may agree with the involvement of SIRT1 in the antiapoptotic effect of BJ and BE, which is able to up‐regulate the expression of SIRT1 and increase its activity. These events are also related to BB prevention of RANKL and sclerostin up‐regulation due to oxidative stress. Thus, the protective effect of BJ and BE is due both to their direct antioxidant action and to the up‐regulation of SIRT1, which does not appear to be a redox‐regulated mechanism. In fact, the expression of SIRT1 does not change in untreated starved cells in the presence of oxidative stress as compared with the control. Indeed, recently it has been demonstrated that SIRT1 overexpression may prevent H_2_O_2_‐induced apoptosis in osteoblast cells by decreasing the activity of caspase‐3 via down‐regulation of the forkhead box O/β‐catenin signalling pathway 51. Many data indicate that the effects of phytocompounds may be due not only to their ROS scavenger activity but also to specific interactions with proteins involved in intracellular signalling pathways related to the regulation of osteoblast and osteoclast activity 30. Indeed, dietary blueberry increased SIRT1 levels in mammals 36, and SIRT1 overexpression has also been related to down‐regulation of sclerostin in ovariectomized female mice 52 and to the inhibition of RANKL‐induced osteoclast differentiation without affecting osteoclast survival 53. Therefore, SIRT1 has been proposed as a potential target for anabolic therapies aiming to block bone resorption and to restore a normal remodelling process. Altogether, these data suggest that the antiapoptotic and antiosteoclastogenic role of BBs in starved MLO‐Y4 cells is due to their antioxidant properties and to SIRT1 activity.

The article "Blueberry juice protects osteocytes and bone precursor cells against oxidative stress partly through SIRT1" was published in 2019. Journal: FEBS Open Bio.

Finally, it has been reported that during tissue regeneration, stem cell proliferation is sensitive to changes of environmental conditions and, in particular, is reduced in the presence of oxidative stress 21, 23.

Thus, our findings on BJ's ability to protect MSCs from damage induced by ROS increase are interesting and worthy of further investigation. Moreover, since metabolites of phenolic acids, derived from vegetable polyphenols, are able to stimulate MSCs versus osteoblast differentiation 23, BJ's effect in MSCs could be related to its polyphenolic components. However, it is noteworthy that in MSCs the highest concentration of TSP does not have a beneficial effect on cell viability, different from what was observed in MLO‐Y4 cells, indicating a possible harmful action in MSCs due to the high concentration of TSP. This may be due to the different sensitivity to the action of BJ of the two types of cells; in fact, MLO‐Y4 cells are highly differentiated and mature osteoblasts, while on the other hand, MSCs are undifferentiated cells and, perhaps, more sensitive either to toxic effects due to oxidative stress or to possible harmful effects of high concentrations of BB phytochemicals. These findings indicate that in the MSCs the beneficial effect of BJ occurs within a certain concentration range of TSP. Moreover, BJ's action in these cells seems to depend in part on SIRT1 activity and this, together with the ability of SIRT1 to promote MSCs' osteogenic differentiation 54, may be very important considering that MSCs are currently considered among the best candidates for cell‐based therapy in regenerative medicine 20, 24. Given that BJ in MSCs does not activate SIRT1 expression, we suggest that its involvement in BJ's protective effect can be due to a post‐translational mechanism(s) in the regulation of SIRT1 activity induced by BJ. It is necessary to further investigate the mechanisms by which SIRT1 in osteocytes as well as in MSCs can contribute to the protective effect of BJ against oxidative stress damage.

The article "Blueberry juice protects osteocytes and bone precursor cells against oxidative stress partly through SIRT1" was published in 2019. Journal: FEBS Open Bio.

## Conclusions

The results of this study demonstrate, for the first time, in osteocytes, cells in close contact with blood capillaries and considered the major regulators of bone remodelling, a significant relationship between the antioxidant activity of BBs and molecular events related to apoptosis and expression of osteoclastogenic factors induced by oxidative stress. Other novel data show that BBs protect MSCs, important cells for bone regeneration, against reduction of viability and cytotoxicity due to oxidative stress. Moreover, the protective effects of BBs both in osteocytes and in MSCs are in part mediated by SIRT1. Indeed, this enzyme is considered a possible target for anti‐resorptive drugs 55 and for anabolic therapies for osteoporosis 52, 53, 56; reduced SIRT1 expression has been associated with osteoporotic hip fracture 57. The present study also reports that two different preparations of BB (juice or extract) containing the same TSP amount show similar effects due to the complex mixture of polyphenols and/or to other bioactive phytochemicals for some of which the bioavailability has been demonstrated 38, 39, 40, 42, 43, 44. This may be interesting, considering that most studies report the effects on bone metabolism of isolated natural compounds, although individuals do not consume isolated molecules but fruits and vegetables rich in many different types of polyphenols and phytochemicals. Overall, these novel data in osteocytes and MSCs may contribute to explain at the cellular and molecular level the protective effects of BB phytochemicals against the damage caused by oxidative stress in bone remodelling and regeneration. Indeed, beneficial anabolic effects of BBs in bone tissue have been reported in animal studies, which suggest blueberries to be a useful supplement for the prevention and/or management of osteoporosis and the osteogenic process 2, 3, 31, 32, 50.

The article "Blueberry juice protects osteocytes and bone precursor cells against oxidative stress partly through SIRT1" was published in 2019. Journal: FEBS Open Bio.

## Materials and methods

### Preparation of blueberry juice and solubilized extracts

BBs, harvested in August 2017/2018 in Tuscany Apennines, were frozen freshly picked in aliquots of 100 g each and used when necessary to prepare BJ by homogenization in a refrigerated Waring blender. The fruit mixture was then filtered under vacuum and centrifuged at 20 000 ***g*** for 10 min to remove insoluble particles. Aliquots of BJ were stored at −20 °C until use. BE was prepared by solubilizing the dry extract, obtained by Aboca SpA (Sansepolcro, Italy), in phosphate‐buffered saline (PBS).

### Determination of total soluble polyphenols

The TSP fraction in BJ and BE was quantified with the Folin–Ciocalteu reagent according to a slightly modified method of Singleton and Rossi using gallic acid as the standard 58. Briefly, 100 μL commercial Folin–Ciocalteu reagent (Merck KGaA, Darmstadt, Germany) diluted 1 : 10 in distilled water was added to 20 μL of sample or standard placed in 96‐well plates. After 5 min, the reaction was stopped by adding 80 μL of saturated Na_2_CO_3_ solution. Samples and standard were kept in the dark at 25 °C for 2 h. Subsequently, the absorbance was measured in a microplate reader at 765 nm. The TSP concentration in BJ, obtained from 100 gr of BB fresh weight, was 1.6 ± 0.1 mg·mL^−1^ (about 50 mg/100 g of fresh weight). TSP concentration in the solution obtained from BB dry extract was 2.3 ± 0.2 mg·mL^−1^ (about 460 mg/100 g of dry extract). In literature, the range of TSP is from 48 to 304 mg/100 g of fresh BB weight 40, and this range strictly depends on the cultivar, growing conditions and maturity, and the estimation may vary depending on the analytical procedure.

### Determination of antioxidant capacity by measuring superoxide anion radical scavenging activity

The antioxidant capacity of BJ and BE, both containing 50 μg·mL^−1^ of TSP, was assayed evaluating the Nitroblue tetrazolium (NBT) reduction mediated by superoxide anion produced by the xanthine/xanthine oxidase system, as previously described 59. Briefly, the superoxide anion, generated by the reaction catalysed by xanthine oxidase in the presence of xanthine, induced the reduction of NBT that represents a target for detection of $O_{2}^{-\cdot }$ scavenging capacity. The coloured reaction, due to the reduction of NBT with the $O_{2}^{-\cdot }$, was detected at 560 nm [Perkin Elmer (Waltham, MA, USA) spectrophotometer]. Antioxidant activity of BJ and BE samples inhibits the colour change. For this assay, reagents used were purchased from Sigma‐Aldrich (St Louis, MO, USA).

The article "Blueberry juice protects osteocytes and bone precursor cells against oxidative stress partly through SIRT1" was published in 2019. Journal: FEBS Open Bio.

### Cell culture and treatment

MLO‐Y4 osteocyte‐like cells (a gift from Dr L. Bonewald, University of Missouri‐Kansas City) were cultured at 37 °C in a 5% CO_2_ humidified atmosphere in α‐MEM supplemented with 5% calf serum (HyClone, GE Healthcare, Chicago, IL, USA), 5% FBS (HyClone, GE Healthcare), 2 mm l‐glutamine, 72 mg·L^−1^ penicillin and 100 mg·mL^−1^ streptomycin (complete medium). MLO‐Y4 cells were grown in complete medium to 70–80% confluence, and then incubated for 1 h in the presence or not of BJ containing TSP at different final concentrations (from 7.5 μg·mL^−1^ to 60 μg·mL^−1^), or in the presence of BE containing TSP at the final concentration of 30 μg·mL^−1^. Subsequently, complete medium was removed, and for another 4 or 24 h the cells were cultured in serum‐free medium (starved cells) in the presence or not of BJ or BE and in fresh complete medium (control). Experiments with EX527 (Sigma‐Aldrich), a specific inhibitor of SIRT1 37, were performed in cells cultured in complete medium in which the inhibitor was added for 30 min at the final concentration of 10 μm. After removing the complete medium, the cells were cultured for another 24 h in serum‐free medium (starved cells) and in fresh complete medium (control) in the presence or not of EX527. Starved cells with or without the inhibitor were treated or not with BJ or BE as reported above.

The MSCs were purchased from ATCC (Manassas, VA, USA), expanded and cultured as previously reported 51. The cells were plated at low density (3–5000 cells·cm^−2^) and incubated for 24 h in 10%, 0.5% or 0.1% or no FBS in the presence or not of BJ at concentrations reported for osteocytes. Experiments with EX527 were performed as previously reported for osteocytes. Some treatments were performed in cells transiently transfected with 75 nm mouse SIRT1 siRNA corresponding to two DNA target sequences of mouse SIRT1 (5′‐GUUACUGCAGGAGUGUAAA[dT][dT]‐3′; 5′‐UUUACACUCCUGCAGUAAC[dT][dT]‐3′) (Sigma‐Aldrich) or scrambled siRNA (Universal Negative Control #1, Sigma‐Aldrich), using Lipofectamine RNAiMAX™ (Invitrogen, Carlsbad, CA, USA) according to the manufacturer's instructions. The ability of siRNA to silence SIRT1 expression levels was checked in control cells 24 h after transfection. In experiments with EX527, 0.008% final concentration of DMSO was present in control and in all treated and untreated cells.

### Determination of intracellular ROS

The intracellular levels of ROS were measured in MLO‐Y4 cells and in MSCs seeded in 12‐well plates and treated with BJ and BE as reported above. One hour before the end of the various treatments, the cell‐permeant probe 2′,7′‐dichlorodihydrofluorescein diacetate (H_2_DCFDA; Invitrogen) was added in culture medium. Once deacetylated by esterases, the probe is rapidly oxidized to a highly fluorescent compound in the presence of ROS. After PBS washing, adherent cells were lysed in RIPA buffer (50 mm Tris/HCL pH 7.5, 1% Triton X‐100, 150 mm NaCl, 100 mm NaF, 2 mm EGTA, phosphatase and protease inhibitor cocktail), centrifuged at 20 000 ***g*** (ALC PK121R, Thermo Fisher Scientific, Waltham, MA, USA) for 10 min, and analysed immediately by fluorescence spectrophotometric analysis at 510 nm. Data were normalized to total protein and expressed as fold‐increase over the control values.

The article "Blueberry juice protects osteocytes and bone precursor cells against oxidative stress partly through SIRT1" was published in 2019. Journal: FEBS Open Bio.

### Cell apoptosis assay

MLO‐Y4 cells, seeded in six‐well plates and treated with BJ and BE, as reported above, were used to assess apoptosis by using Cell Death Detection ELISAplus Kit (Roche Laboratories, Nutley, NJ, USA), and annexin V–FITC Kit (Miltenyl Biotec GmbH, Bergisch Gladbach, Germany), according to the manufacturer's instructions. The specific increase of mono‐ and oligonucleosomes released by 10^4^ cells in the cytoplasmic fractions was detected, and data are expressed as fold‐increase over the control values using the following ratio: absorbance of the sample/absorbance of the control values. Cells treated with annexin V–FITC were analysed using a flow cytometer (FACSCalibur; BD Biosciences, San Jose, CA, USA). cellquest™ software (version 3.3; BD Biosciences) was used for analysis relative to the phosphatidylserine present outside the plasma membranes and data are expressed as fold‐increase over the control values.

### Cell viability and cytotoxicity assays

The MSCs were incubated for 24 h in DMEM containing 10% FBS in the absence or in the presence of compounds as reported above. Oxidative stress was induced by reduction of serum in the culture medium. Cell viability was evaluated by non‐radioactive cell assay (MTT) (CellTiter 96^®^ Assay; Promega Corp., Madison, WI, USA) according to the manufacturer's instructions and as previously reported 60, 61. Cell cytotoxicity was determined by using CytoTox 96^®^ Non‐Radioactive Cytotoxicity Assay (Promega), a colorimetric assay that measures lactate dehydrogenase, a stable cytosolic enzyme that is released upon cell lysis. Apoptotic cell fraction was determined after fixation and propidium iodide staining by TALI^®^ cytometry (Life Technologies, Carlsbad, CA, USA) 61.

### Western blot analysis

The phosphorylation of ERK1/2 and JNK, and the expression of activated caspase‐3, PARP‐1, SIRT1, RANKL, sclerostin and Ac‐p53 were performed by western blot in MLO‐Y4 cells seeded in 60 mm tissue culture dish treated as reported above. Cells were lysed for 30 min at 4 °C in ice‐cold RIPA buffer and centrifuged at 20 000 ***g*** for 10 min. Equal amounts of total proteins (40–60 μg) were loaded in each line and were subjected to SDS/PAGE on 10% gel and electrotransferred to poly(vinylidene difluoride) membrane (GE Healthcare). Membranes were probed with specific primary antibody anti‐caspase‐3 or anti‐phospho‐ERK1/2 or anti‐phospho‐JNK or anti‐PARP‐1 (Cell Signalling Technology, Danvers, MA, USA) or anti‐SIRT1 or anti‐RANKL or anti‐sclerostin (Santa Cruz Biotechnology, Inc., Dallas, TX, USA), or anti‐Ac‐p53 (Thermo Fisher Scientific). Subsequently, after stripping the membranes were reprobed with anti‐ERK1/2 or anti‐JNK or anti‐β‐actin for normalization of densitometric values. Secondary antibodies conjugated to horseradish peroxidase were used to detect antigen–antibody complexes using a chemiluminescence reagent kit (Clarity Western ECL Substrate, Bio‐Rad, Hercules, CA, USA). imagej software (National Institutes of Health, Bethesda, MD, USA) was used to perform quantitative analyses, and the values of the bands were expressed as fold‐increase relative to control values.

The article "Blueberry juice protects osteocytes and bone precursor cells against oxidative stress partly through SIRT1" was published in 2019. Journal: FEBS Open Bio.

### Protein assay

Protein concentrations were determined by the bicinchoninic acid solution protein reagent assay (Thermo Fisher Scientific) using bovine serum albumin as the standard (Sigma‐Aldrich).

### Statistical analysis

Each experiment was performed a minimum of three times. Data are expressed as means ± SEM and statistical significance was determined by one‐way ANOVA with Bonferroni's multiple comparison test, using prism software (GraphPad Software Inc., La Jolla, CA, USA). *P* ≤ 0.05 was considered statistically significant.

## Conflict of interest

The authors declare no conflict of interest.

## Author contributions

CG, EM, TI, MLB, and MTV designed the experiments and analysed the data. VD, GM, FP, and LCM performed the experiments. GB performed the apoptosis experiments with the annexin V–FITC kit. VD, EM, TI, and MTV wrote the manuscript.
